The article "Study on the Grading Model of Hepatic Steatosis Based on Improved DenseNet" was published in 2022. Journal: J Healthc Eng.

# Study on the Grading Model of Hepatic Steatosis Based on Improved DenseNet

**DOI:** 10.1155/2022/9601470

**Published:** 2022-03-17

**Authors:** Ruwen Yang, Yaru Zhou, Weiwei Liu, Hongtao Shang

**Affiliations:** ^1^First Clinical Medical College, Nanjing University of Chinese Medicine, Nanjing 210004, China; ^2^Affiliated Hospital, Nanjing University of Chinese Medicine, Nanjing 210004, China

## Abstract

To achieve intelligent grading of hepatic steatosis, a deep learning-based method for grading hepatic steatosis was proposed by introducing migration learning in the DenseNet model, and the effectiveness of the method was verified by applying it to the practice of grading hepatic steatosis. The results show that the proposed method can significantly reduce the number of model iterations and improve the model convergence speed and prediction accuracy by introducing migration learning in the deep learning DenseNet model, with an accuracy of more than 85%, sensitivity of more than 94%, specificity of about 80%, and good prediction performance on the training and test sets. It can also detect hepatic steatosis grade 1 more accurately and reliably, and achieve automated and more accurate grading, which has some practical application value.

## 1. Introduction

The liver, as an important organ of the body, is the key to regulating lipid metabolism in the body. When the body's lipid metabolism is abnormal, it will lead to lipid accumulation in the liver and liver steatosis. Severe liver steatosis is irreversible and threatens human life and health, while milder liver steatosis can be completely cured by treatment. Therefore, early screening for hepatic steatosis is of clinical importance. At present, the degree of hepatic steatosis is mainly determined by manual grading, in which the imaging physician analyzes the patient's imaging data to score the grade of hepatic steatosis. This approach suffers from subjective grading bias and low efficiency. In recent years, with the widespread use of deep learning in medicine, new opportunities for intelligent grading of hepatic steatosis have been presented. For example, Qiblawey Yazan and Montalbo Francis Jesmar P. proposed a cascade system to detect, localize, and quantify COVID-19 infection from CT images using encoder-decoder convolutional neural networks (ED-CNNs), UNet, and feature pyramid network (FPN) [1, 2]. Ben Jabra Marwa used 16 deep learning classifiers to diagnose the validity of COVID-19 from chest X-ray images and found that the combination of deep learning models and integrated classification techniques resulted in the highest confidence level for class 3 classification [3]. Liu Zhenguo et al. identified patients with myasthenia gravis effectively based on the 3D DenseNet deep learning (DL) model of preoperative CT of patients as a complement to the conventional diagnostic criteria for identifying thymoma-associated MG [4]. Riasatian Abtin et al. used a DenseNet topology with four dense blocks, fine tuned and trained with different structures to propose a KimiaNet histopathology image recognition model, and tested KimiaNet using three publicly available datasets of TCGA, endometrial cancer images, and colorectal cancer images to verify the effectiveness of the model [5]. The model has certain search and classification performance when used for image representation. Considering the correlation of multilead ECG, systematically mining the correlation of interlead signals, and enhancing the multiplexing of feature information between interlead and intralead signals by using the dense connection of DenseNet, Xiong Peng et al. proposed a novel multilead myocardial infarction localization method based on a densely connected convolutional network (DenseNet), which automatically captures valid myocardial infarction, improves its recognition rate, and can be introduced into clinical practice to assist in the diagnosis of myocardial infarction [6]. Albahli Saleh et al. proposed three different BiT models: the DenseNet, InceptionV3, and Inception-ReNetV4 for the diagnosis of coronavirus pneumonia patients by X-ray chest radiographs, and the results showed that the pretrained DenseNet model had the highest classification efficiency of 92%, the accuracy of Inception V3 was 83.47% and that of Inception-ResNetV4 was 85.57%. This is sufficient to show the advantages of the DenseNet algorithm [7]. Wang Gaihua et al. proposed an image classification model with a residual attention mechanism based on the improved DenseNet, extracting image features from the training set, which can improve the accuracy of DenseNet algorithm by 8.89% [8]. It can be seen that deep learning has been effective in identifying various diseases in medicine, and it has certain auxiliary functions for physicians to diagnose diseases. Therefore, based on the above research studies, this paper combines the DenseNet algorithm of deep learning with transfer learning to propose a migration learning-based method for grading hepatic steatosis with the improved DenseNet model.

The article "Study on the Grading Model of Hepatic Steatosis Based on Improved DenseNet" was published in 2022. Journal: J Healthc Eng.

## 2. Basic Methods

### 2.1. Introduction to DenseNet Algorithm

The DenseNet algorithm is a neural network that uses feature combinations and set bypasses to improve the performance of the network, which enables the summation of the features of the two pathways before and after the block by means of dense connections [9], which in turn improves the reuse of the features by the network. One *L*-layer DenseNet network includes *L*(*L* + 1)/2 connections to ensure that model short-circuit values occur in blocks. However, to ensure no short circuiting between blocks, the model adds a pooling layer to approximately reduce the parameters, while ensuring a relatively small model size. The DenseNet model block is shown in Figure 1. The input of layer *i* is *X*_*t*_, which can be expressed as

(1) $$\begin{array}{c} X_{t}=H_{t}\left(\left[X_{0},X_{1},...,X_{t-1}\right]\right) \end{array}$$

where *H* is the nonlinear transform, usually a combination of BN + ReLU + Conv(3*∗*3); *X*_0_ and *X*_*t*−1_ are all layers before the *i*-th layer; is the stitching, indicating that all outputs from *X*_0_ to *X*_*t*−1_ are stitched.

#### 2.1.1. DenseNet Algorithm Improvements

The DenseNet model extracts features by training from scratch, which tends to lead the model fall into local optimum. In addition, to obtain the best prediction, the model often needs a large amount of data support, which leads to a deepening network, and a too deep network will reduce the learning ability of the model, which in turn is prone to overfitting. At the same time, the radio image used for liver steatosis grading is usually small compared to conventional image datasets so that the model is less effective in classification recognition. To solve the above problems, the DenseNet model is improved in this paper. According to the literature [10, 11], if two domains have commonality, their “knowledge” can be transferred; i.e., the knowledge learned from one domain can be used in the other domain. Therefore, this paper improves the DenseNet model by combining transfer learning. In this paper, we improve the training accuracy of the model by transferring the pretrained model from the world's largest image recognition library (ImageNet dataset) into the DenseNet model [12].

When training a DenseNet model based on transfer learning, the amount of data (batch-size) fed into each iteration is only a small fraction of all the data, and the larger the batch-size, the less time it takes to train the model for one round (epoch). After increasing the batch size *n* times, the time per batch is $\sqrt{\text{n}}$. Considering the existence of a local minimum in the design training, the objective of the training is to minimize the softmax function. During the training process, the learning rate determines the update step of the iterations, and if its value is too large, it tends to cause the loss function not to converge, too small to fall more slowly. The best value can be selected by observation.

The regular model gradient descent update weight is as follows [13]:

(2) $$\begin{array}{c} w^{\prime }=w-a\cdot \nabla c, \end{array}$$

where *w*′ and *w* denote the connection weights after and before the update, *a* denotes the learning rate, and ∇*c* denotes the backpropagation gradient. After adding the momentum, the above equation can be rewritten as

(3) $$\begin{array}{c} v^{\prime }=\text{momentum}\cdot v-a\cdot \nabla c, \end{array}$$

(4) $$\begin{array}{c} w^{\prime }=w+v^{\prime }, \end{array}$$

where *v* denotes the iterative gradient cumulative information and momentum is the momentum coefficient, which usually takes the value of 0.9 to 0.99 [14].

The article "Study on the Grading Model of Hepatic Steatosis Based on Improved DenseNet" was published in 2022. Journal: J Healthc Eng.

## 3. Deep Learning for Liver Steatosis Grading Practice

Based on the above analysis of the DenseNet model related to transfer learning, the specific method of using deep learning for liver steatosis grading study in this paper is as follows:

1. Dataset construction. All patients' clinical information is concealed, the grade of hepatic steatosis is labeled and used as a tag, and the dataset with their corresponding ROI is constituted.
2. Data preprocessing. To improve the convergence speed of the network, the datasets are dealed with normalization, the patient MRI image pixels are normalized to [0, 1] without changing the stored information of images, and the training set and test set are divided in a certain ratio [15].
3. Model construction and training. Based on the basic structure of DenseNet, a DenseNet model is built and transfer learning feedforward and backpropagation algorithms are trained on low-level weights and high-level weights, respectively, to identify the features of the discovered structures and specific images in the images. In this paper, 1.28 million natural images from the ImageNet dataset are selected for pretraining the model.
4. Model fine tuning. Model fine tuning usually includes by training the whole network, freezing the convolutional base, and freezing some layers to train some layers [16]. Considering the difference in data volume between the experimental dataset and the ImageNet dataset on the hepatic steatosis study in this paper, it was decided to choose the approach of freezing some layers to train some layers for model fine tuning[17]. After the model is pretrained, the fully connected layer is removed, 2 dense blocks are frozen, and 1 untrained dense block and the fully connected layer are added immediately afterwards, with the aim of extracting and classifying advanced features, which then connected by batch normalization and pooling layers [18]. Ultimately, the model structure used in this paper for liver steatosis grading study is shown in Figure 2. In the figure, Dense Block1, Dense Block2, and Dense Block3 are densely connected in 4, 4, and 32 layers, respectively.

The article "Study on the Grading Model of Hepatic Steatosis Based on Improved DenseNet" was published in 2022. Journal: J Healthc Eng.

## 4. Simulation Experiments

### 4.1. Experimental Environment Setup

The experiments were conducted on an Nvidia GeForce RTX 2080 Ti GPU, implemented through the Keras deep learning framework, and programmed in Python 3.6.

### 4.2. Data Source and Preprocessing

The data of this experiment were obtained from abdominal MR imaging data and clinical information of 50 patients from June to July 2020 in a hospital in Beijing. Among them, hepatic fat grade grading was done independently by two professional imaging physicians based on patient imaging data, and hepatocellular steatosis was divided into four degree scores, noting hepatocellular adipocyte deformation 0–5% as 0, 5–33% as 1, 34%–66% as 2, and more than 66% as 3, respectively [19]. The statistics of patients' hepatic steatosis grade shows that there were 38 patients with grade 0, 24 male patients and 14 female patients; 12 patients with grade 1, 6 male patients and 1 female patient; there were no patients with grade 2 or 3.

Figure 2 shows an example of an MR abdominal mDixon imaging slice of a patient. Six square ROI regions were set for each MR sequence of DICOM images under the premise of avoiding large blood vessels, focal liver lesions, and significant liver artifacts [20]. Four of the ROIs were located in the parenchyma of the right lobe of the patient's liver, i.e., segments V, VI, VII, and VIII of the liver, and the other two ROIs were located in the parenchyma of the left lobe of the patient's liver, i.e., segments II and III of the liver. Each region of the liver parenchyma has 16*∗*16 pixels.

Considering the small amount of experimental data, only 300 ROIs of 50 patients, it is difficult to meet the demand of deep learning data volume, so the experiment uses panning, rotation, mirroring, and other enhancement processing on the data [21]. In addition, since the difference in the number of data between samples with liver fat deformation as grade 0 (38 cases) and grade 1 (12 cases) is more obvious, if directly input into the depth model, it will easily lead to the neglect of the minority class samples, which are of important research value in medical image analysis. Therefore, to avoid the effect of unbalanced data samples on the results, the experiments combined the actual number of minority class samples and majority class samples and used the method of oversampling minority class samples to deal with unbalanced data samples [22, 23]. The 648 ROIs with grade 1 hepatic steatosis were amplified twice with 2-fold data to obtain a total of 2,592 cases of grade 1 hepatic steatosis ROI data. Finally, 2,052 cases of grade 0 ROI data and 2,592 cases of grade 1 ROI data of hepatic steatosis were obtained in this experiment, where 3,766 and 878 ROIs were used for model training and testing, respectively, and Adam was selected as the optimization algorithm during the modeling process.

The article "Study on the Grading Model of Hepatic Steatosis Based on Improved DenseNet" was published in 2022. Journal: J Healthc Eng.

### 4.3. Evaluation Indexes

In this experiment, precision, sensitivity, specificity, and AUC were chosen as the indexes to evaluate the model performance. Precision reflects the probability that the model predicts correctly for all samples and is calculated as in equation (5). Sensitivity is a measure of the probability that the model predicts correctly for positive class samples and is calculated as in equation (6). The specificity is a measure of the probability that the model correctly predicts the negative class samples and is calculated as in equation (7). The higher the values of precision, sensitivity, and specificity, the better the model performance. AUC, the probability of predicting a positive case before a negative case, is an important index of the predictive effectiveness of a dichotomous classification model. The closer its value is to 1, the better the model performance is indicated [24].

(5) $$\begin{array}{c} \text{precision}=\frac{TP}{\left(TP+FP\right)}, \end{array}$$

(6) $$\begin{array}{c} \text{sensitivity}=\frac{TP}{P}, \end{array}$$

(7) $$\begin{array}{c} \text{specificity}=\frac{TN}{N}, \end{array}$$

where *TP* denotes true positive; *FP* denotes false positive; *P* denotes all positive; *TN* denotes true negative; *N* denotes all negative. The accuracy and the loss function were selected to evaluate the metrics for evaluating the change of the model during training and testing. The accuracy rate reflects the probability of correct prediction during the model iteration and is calculated as in equation (8). The closer its value is to 1, the higher the model prediction accuracy is. The loss function reflects the difference between the predicted label and the true label, and is calculated as in equation (9). The closer its value is to 0, the better the model prediction is, and the closer the predicted value is to the true value [25].

(8) $$\begin{array}{c} \text{accuracy}=\frac{TP+TN}{P+N}, \end{array}$$

(9) $$\begin{array}{c} \text{loss}=\left[y\;\log\;\hat{y}+\left(1+y\right)\text{log}\left(1-\hat{y}\right)\right]. \end{array}$$

In equation (9), *y* and $\hat{y}$ denote the true label and the predicted label, respectively.

### 4.4. Experimental Results

#### 4.4.1. Model Validation

To verify the effectiveness of the proposed model transfer learning for model improvement, the experiments compare the training error of the model before and after the transfer learning with the test set accuracy, and the results are shown in Figure 3, where a and *b* are the model training error and test set accuracy before transfer learning, with the number of iterations, respectively, and *c* and *d* are the model training error and test set accuracy after transfer learning, with the number of iterations, respectively. As can be seen from the figure, before transfer learning, the model reached convergence at about 100,000 iterations and its accuracy on the test set was 80%; after transfer learning, the model converged at about 30,000 iterations and its accuracy on the test set was 83.4%. It shows that transfer learning can improve the model convergence speed and prediction accuracy.

The article "Study on the Grading Model of Hepatic Steatosis Based on Improved DenseNet" was published in 2022. Journal: J Healthc Eng.

To further validate the effectiveness of transfer learning, the confusion matrix of the model's prediction of each grade of hepatic steatosis after transfer learning was experimentally analyzed, as shown in Figure 4, where the horizontal and vertical coordinates are the sample prediction and the true grade, respectively, and the diagonal line is the proportion of correct predictions. As can be seen from the figure, the proposed model has a high accuracy in predicting the grade of hepatic steatosis, which is more than 80%.

In addition, the experiments also compared the prediction effects of the proposed model with other models before and after transfer learning, and the results are shown in Table 1. As can be seen from the table, the accuracy of the model after transfer learning is improved in different degrees on the test set compared with the model before transfer learning; the proposed model has a higher accuracy of 83% on the test set compared with other transfer learning models, and the smaller the model size is, the shorter the time to predict a single image, which shows that the proposed model has certain superiority.

#### 4.4.2. Model Prediction Results

To verify the validity of the proposed model for liver steatosis grading practice, the accuracy, sensitivity, specificity, and AUC values of the model on the training and test sets were collected experimentally, and the results are shown in Table 2. As shown in the table, the accuracy of the model on the training and test sets was more than 85%, the sensitivity was more than 94%, the specificity was about 80%, and the AUC value was more than 0.8, which is closer to 1. This indicates that the proposed model has good predictive performance and can predict the grade of hepatic steatosis of patients more accurately. The sensitivity and specificity indicate that the model has a strong ability to detect positive cases, indicating that the model can detect hepatic steatosis grade 1 more reliably and has some practical application value.

The article "Study on the Grading Model of Hepatic Steatosis Based on Improved DenseNet" was published in 2022. Journal: J Healthc Eng.

Figure 5 shows the changes of loss and accuracy curves on the training and testing sets during the iterations of the model. From the figure, it can be seen that with the increase of iterations, the loss and accuracy curves gradually leveled off and reached a stable state after 400 iterations; the model did not show any overfitting phenomenon during the whole training and testing process, which indicates that the proposed model exhibits good prediction performance through transfer learning.

#### 4.4.3. Statistical Analysis

Spielman correlation analysis was performed using MATLAB R2018b on the obtained clinical information, such as gender and age of the patients, and the grade of hepatic steatosis, and the results are shown in Table 3, where *P* < 0.05 indicates a statistically significant difference, and *∗* indicates a significant correlation at the 0.05 level. The table shows that the *p* value of pancreatic steatosis grade and hepatic steatosis grade was 0.003, and the correlation between them was significant; the *p* value of other clinical information such as patient age and gender and hepatic steatosis grade was larger than 0.05, indicating that the correlation between them was not significant.

Correlation analysis between clinical information and hepatic steatosis grade in patients of different genders revealed significant correlations between hepatic steatosis grade and metabolic syndrome and pancreatic steatosis grade in female patients *P* = 0.007 and *P* = 0.002, while there was no correlation between hepatic steatosis grade and its clinical information in male patients. The change in liver fat content with age of the patients was analyzed, and the results are shown in Figure 6. As can be seen from the figure, there was no correlation between liver fat content and the age of the patients, but there was a peak between the ages of 50 and 60 years for women and one peak each between the ages of 40 and 50 years and 70 to 80 years for men.

## 5. Conclusion

In summary, applying deep learning to liver steatosis time can achieve automated and more accurate grading, and by introducing transfer learning into the deep learning DenseNet model, the number of model iterations can be significantly reduced and the model convergence speed and prediction accuracy can be improved, which has some potential application value. Applying it to the practice of liver steatosis grading, the accuracy of the proposed model on the training and test sets reached more than 85%, the sensitivity exceeded 94%, the specificity was about 80%, and the AUC value reached more than 0.8, which is closer to 1. It has good predictive performance and can detect liver steatosis grade 1 more accurately and reliably, which has some practical application value. Statistical correlation analysis shows that hepatic steatosis correlates significantly with pancreatic steatosis and has some correlation with metabolic syndrome; hepatic steatosis was correlated with age and metabolic syndrome in women only. However, due to the limitations, there are still some shortcomings in this paper; the amount of patient data is too small, the preliminary results obtained need to be further validated, and among the 50 patients with hepatic steatosis, there are no patients with grade 1 or higher, which leads to the accuracy and generalization ability of the model to be demonstrated. Therefore, the amount of hepatic steatosis imaging data will be further collected and expanded in the next study.

The article "Study on the Grading Model of Hepatic Steatosis Based on Improved DenseNet" was published in 2022. Journal: J Healthc Eng.

## Figures and Tables

**Figure 1:** Dense connection of DenseNet blocks.

**Figure 2:** Example of mDixon slice image.

**Figure 3:** Performance comparison before and after model transfer learning.

**Figure 4:** Confusion matrix of model prediction results.

**Figure 5:** Model performance iteration curve.

**Figure 6:** Variation curve of liver fat content with age.

**Table 1:** Comparison of prediction results of different models.

Network name	Testing set accuracy		Model size (MB)	The time of predicting single image(s)
	Nontransferable learning (%)	Transfer learning (%)		
ResNet52	68.34	70.33	235	0.2447
VGG16	77.25	79.48	521	0.0630
VGG19	77.31	80.27	561	0.0704
SqueezeNet	73.09	77.36	2.77	0.0072
GoogleNet-inception V1	78.42	80.46	39.4	0.0221
DenseNet 16	80.27	83.46	101	0.2721

**Table 2:** Model performance.

Items	Accuracy (%)	Sensitivity (%)	Specificity (%)
Training sets	88.49	95.44	81.6
Test sets	85.79	94.55	79.82

**Table 3:** Analysis results of clinical information and hepatic steatosis grade of patients.

Clinical information	Correlation coefficient	*P* value
Age	0.003	0.959
Gender	0.035	0.570
Pancreatic steatosis grade	0.702*∗*	0.003
Metabolic syndrome	0.890	0.147

## Data Availability

The experimental data used to support the findings of this study are available from the corresponding author upon request.
